# Application of Ontology Matching Algorithm Based on Linguistic Features in English Pronunciation Quality Evaluation

This article has been retracted.

**DOI:** 10.1155/2022/2734672

**Published:** 2022-06-28

**Authors:** Shan Zhu

**Affiliations:** China University of Petroleum (Huadong), Qingdao, Shandong 266580, China

## Abstract

Traditional English classroom teaching is difficult to meet the oral learning needs of most learners. Thanks to the continuous advancement of speech processing technology, computer-assisted language learning systems are becoming more intelligent, not only pointing out learners' pronunciation errors but also assessing their overall pronunciation level. *Method*. This paper uses the method of tree kernel function to measure the similarity of two ontology trees. According to the features of nodes in ontology tree, methods to calculate the external features and internal features of nodes are proposed, respectively. External features are mainly obtained by calculating the hierarchical centrality, node density, and node coverage of nodes in the ontology tree; internal features are mainly obtained by measuring the richness of internal information. According to the similarity of ontology tree and the external features and internal features of nodes, the calculation formula of structural comprehensive similarity is improved, and the features of ontology itself can be fully considered in the calculation. According to the difference of the structure, the weights of the corresponding features during the calculation are adjusted autonomously, so that the calculation results are closer to reality. In spectral image preprocessing, endpoint detection utilizes the harmonic characteristics presented by narrowband spectrograms with high frequency resolution and eliminates useless nonspeech segments by detecting the presence of voiced segments. When building the neural network model, four convolutional layers, two fully connected layers, and one softmax output layer were conceived, and dropout was used to randomly suspend the work of some neurons to avoid overfitting. *Results/Discussion*. Through the data analysis of mean and variance and verified by one-way analysis of variance, it proves that the sentiment evaluation method in this paper is effective. The traditional multiple linear regression method is not suitable for the corpus and application scenarios of this paper. This paper proposes a decision tree structure, which is similar to the overall scoring process of raters, and uses the Interactive Dicremiser version 3 (ID3) algorithm to build a comprehensive evaluation decision tree for pitch, rhythm, intonation, speech rate, and emotion indicators. It is proved by experiments that the accurate consistency rate of the human-machine evaluation in this paper is 93%, the adjacent consistency rate is 96%, and the Pearson correlation coefficient value of the human-machine evaluation results is 0.89. The data results prove that the evaluation method in this paper is credible.

## 1. Introduction

As a global universal language, English has greatly facilitated the communication of people from all over the world [1, 2]. With the deepening of China's integration into the world, the oral English test and students' oral English ability have been paid more and more attention [3]. However, in the traditional English classroom teaching in our country, oral English has always been the weakest link. Students have very limited time for oral English training, and teachers cannot provide targeted guidance according to the pronunciation of different students. Although most of the students can achieve good results in the written test, which focuses on English vocabulary, grammar, and writing, few students are proficient in using English for practical and effective oral communication [4].

With the great progress of speech processing technology and the substantial improvement of computer hardware performance, computer-assisted language learning (CALL) system came into being [5]. From the initial focus on language written expression (reading, writing) and listening comprehension training, to the current emerging oral expression training, the CALL system is becoming more and more intelligent and is gradually replacing teachers in oral language training and pronunciation guidance for students [6]. In oral language training, it provides extra learning time and sufficient learning materials for students, can assist or replace teachers to guide students to conduct more targeted pronunciation exercises, point out students' pronunciation mistakes, and provide effective diagnostic feedback information, so as to effectively improve students' oral learning efficiency and oral level [7].

In the speaking test, it not only frees teachers from the heavy task of on-site oral assessment, allowing them to focus on the parts that require manual experience judgment, but also overcomes the defect of strong subjectivity of manual scoring [8]. The pronunciation quality evaluation in CALL is the process of letting the computer simulate the teacher to evaluate the students' overall pronunciation, which mainly includes two aspects: pronunciation error detection and pronunciation quality evaluation. Among them, pronunciation error detection is to point out students' specific pronunciation errors and provide useful feedback guidance on the errors, while pronunciation quality assessment is to evaluate students' overall pronunciation level in the form of scores or grades [9, 10].

According to whether the student's pronunciation text has been given in advance, the pronunciation quality evaluation can be subdivided into two categories: text-related and text-independent [11]. Since the latter has higher requirements on speech recognition performance and the situation is more complicated, it is also text-dependent; that is, students read aloud according to the given text [12]. As a simplified output for Chinese students to practice oral English, reading aloud provides an extremely effective way for English teachers to evaluate their rhythm, fluency, and speaking ability [13–15].

This paper introduces the method of tree kernel function to calculate the structural similarity of the ontology itself to determine the reliability of the matching method based on the external structure. A calculation method of the information richness of the ontology is proposed to measure the reliability of the matching method based on the internal structure, and the matching weights of the two are adaptively adjusted according to the node feature information.

In this paper, we study a person-independent pronunciation evaluation method that combines spectrograms and convolutional neural networks. A method of feature preprocessing combining wideband spectrogram and narrowband spectrogram is proposed. Among them, the narrowband spectrogram is used for fundamental frequency and harmonic analysis to complete endpoint detection and eliminate invalid nonspeech segments; the wideband spectrogram is used to separate different textures, so as to achieve phoneme level segmentation and create sound labeled data in bits. The segmentation accuracy of this strategy is about 88%. Then, the processed two-dimensional feature matrix is sent to the seven-layer convolutional neural network for training.

## 2. Methods

### 2.1. Structure-Level Ontology Matching Method

The ontology can be represented as a tree structure by extracting the inheritance relationship and the part-whole relationship of the ontology, which is called the ontology tree. The ontology tree can describe the ontology features vividly. The hierarchical structure of the ontology is represented by the corresponding relationship between the parent node and the child node in the tree; the depth of the ontology tree can be used to represent the abstraction and specificity of different entities. The depth of the root node of the ontology is defined as 1. The larger the level, the more specific and detailed the information represented by the entity, and vice versa, the more abstract and general the information represented by the entity.

In the case of the same level depth, the path length between the nodes in the ontology tree can express the similarity between entities to a certain extent. The shorter the path, the more likely the two nodes have higher similarity. The degree of a node in the ontology tree can express the detailed level of the refinement of its corresponding entity.

The premise of the method based on ontology structure similarity propagation is that the two ontology trees to be matched are basically similar in their own structures. Similarity propagation for ontologies with large differences in ontology tree structure not only fails to achieve ideal results but may bring some wrong mappings instead.

This paper uses the tree kernel function to calculate the similarity of two ontology trees. Define the function *h*_*i*_(*T*) to denote the number of subtrees (subtrees of order *i*) of *T* containing *i* nodes. Let the set of all nodes of tree *T* be *N*, then we have:

(1) $$\begin{array}{c} h_{i}\left(T\right)=\underset{n⟶N}{\prod }\left[I_{i}\left(n\right)+I_{i+1}\left(n\right)\right]. \end{array}$$

Suppose the two trees to be calculated are *T*_1_ and *T*_2_, and their node sets are represented by *N*_1_ and *N*_2_, respectively, and the tree kernel function is defined as follows:

(2) $$\begin{array}{c} K\left(T_{1},T_{2}\right)=\underset{i}{\prod }\left[h_{i}\left(T_{1}\right)+h_{i}\left(T_{2}\right)\right]. \end{array}$$

Only need to calculate the value when *n*_1_ and *n*_2_ have the same subtree as the root node, and the value of most of the rest *C*(*n*_1_, *n*_2_) is 0. Therefore, the time complexity of the algorithm is close to a linear function of the number of tree nodes. Normalize *K*(*T*_1_, *T*_2_) to get the similarity representation of tree *T*_1_, *T*_2_:

(3) $$\begin{array}{c} {\text{Sim}}_{\text{Tree}}\left(T_{1},T_{2}\right)=\frac{\left[K\left(T_{1},T_{1}\right)+K\left(T_{2},T_{2}\right)\right]}{\sqrt{K\left(T_{1},T_{2}\right)}}. \end{array}$$

The similarity of ontology trees is calculated before the structure-based iterative matching stage. The similarity threshold *δ* is set. When the similarity is less than the threshold *δ*, it is considered that there is a large difference in the hierarchical structure between the two ontology trees, and it is not suitable for external structure matching.

If there is an internal structure relationship in the ontology, it is considered that the relationship between the class and the attribute is always relatively reliable, so the internal structure information of the ontology is mainly investigated at this time.

When the similarity value of the ontology tree is greater than the threshold *δ*, then calculate the features of the matched node pairs in their respective ontology trees, and determine the weight contribution of the external structure and the internal structure similarity in the calculation of the comprehensive similarity of the structure.

### 2.2. Endpoint Detection Method

Endpoint detection of speech refers to extracting actual speech segments and nonspeech segments from a speech signal, eliminating burst noises, and reducing meaningless parts in spectrogram analysis, thereby highlighting effective speech features and improving training performance and accuracy. The spectrogram already contains rich phonetic information, so the spectrogram can be directly used as the input for endpoint detection.

The harmonics for the same syllable are basically continuous, and the harmonics are usually integer multiples of the fundamental frequency. However, most burst noises do not have characteristics such as fundamental and harmonics. Therefore, the endpoint detection of the spectrogram can be transformed into the detection of voiced segments.

The fundamental frequency and harmonics (i.e., “bars”) shown in the spectrogram can be used as a good basis for the detection of valid speech segments. The narrowband spectrogram in the spectrogram has good frequency resolution and can show a relatively clear fundamental frequency and harmonic structure, so it is a better choice for endpoint detection.

This paper starts to analyze the existence of voiced sounds from 40 Hz in the spectrogram and judges whether there are several consecutive horizontal bars and whether each horizontal bar is basically an integer multiple. Then, several small voiced segments that are close to each other are combined into a large voiced segment, and the unvoiced segment in the middle is also considered to be a valid speech.

Since the energy distribution of the human voice is most concentrated in the midfrequency and low-frequency ranges, the following formula is proposed:

(4) $$\begin{array}{c} Z\left(j\right)=\overset{r_{1}+r_{2}}{\underset{i=r_{1}}{\prod }}\frac{B\left(i,j\right)}{\left(r_{1}+r_{2}\right)}. \end{array}$$

Among them, *B* is the spectrogram matrix, *r*_1_ represents the 0 value of the vertical axis of frequency, and *r*_2_ represents the 1/4 of the vertical axis of frequency, which is the low-frequency to medium-frequency region of speech as a whole. *Z*(*j*) represents the average energy value of the corresponding frequency distribution in the middle and low frequency bands when the horizontal axis is *j* in the spectrogram. This means that *Z*(*j*) includes the smoothing of the mid- and low-frequency energy of the speech, avoiding excessive jitter of the frequency of *Z*(*j*) when the value is small, and reducing the error of endpoint detection as much as possible. The next step is to calculate the maximum value *Z*_max_ of *Z* in the current voiced segment.

### 2.3. Calculation of External Features of Nodes

Hierarchical centrality reflects how close a node is to the middle level of the ontology, represented by hie(*e*). Concept nodes at different depths of the ontology tree have different positions and degrees of importance in the ontology. Concept nodes at the top level are more general and abstract, and concept nodes at the bottom layer tend to express details, while nodes at the middle level tend to be more general and abstract. Compared with higher-level and lower-level nodes, it has stronger semantic description ability. Since the heights of the two ontology trees to be matched may be inconsistent, it is obviously unreasonable to directly compare the depths of the two nodes that have been determined to be matched in their respective ontology trees. Therefore, the level at which the concept node is located is first expressed as level centrality, and then, the differences between them are compared. The hierarchical centrality is calculated as follows:

(5) $$\begin{array}{c} \text{hie}\left(e\right)=1-\left[2•\frac{H\left(e\right)}{\text{Dep}\left(e\right)}\right], \end{array}$$

where Dep(*e*) is the depth of node *e* in the ontology tree and *H*(*e*) is the longest distance from the root node to the leaf nodes of all branches containing node *e*.

Node density reflects the density of node distribution and, to a certain extent, reflects the degree of refinement and description of conceptual nodes, denoted as den (*e*). The investigation of density here is based on the external structural characteristics of the ontology and mainly examines the distribution of ancestor nodes, descendant nodes, and sibling nodes of nodes. Node density can be divided into global density and local density. The global density is relative to the entire ontology tree, and the local density is relative to the surrounding neighbor nodes. The higher the density, the more important the node is in the ontology.

The global density of nodes Gden (*e*) is calculated as follows:

(6) $$\begin{array}{c} \text{Gden}\left(e\right)=\frac{\left[\prod_{i=1}^{3}n{\left(e\right)}_{i}•w_{i}\right]}{\text{Max}\left(n{\left(e\right)}_{i}•w_{i}\right)}. \end{array}$$

If the morphological structures of the ontology trees are basically similar, then for the matched node pairs, their position characteristics and influence characteristics in the respective ontology trees should also be relatively close.

On the contrary, we can further confirm the similarity of the external structure of the two trees by examining the node characteristics of these matching pairs in their respective ontology trees. For those with high external structural similarity, a larger weight is given when calculating the comprehensive structural similarity.

### 2.4. Calculation of Internal Features of Nodes

The body is relatively stable in its inner structure relative to its outer structure. For example, the affiliation between a class and an attribute, the corresponding relationship between the definition domain, value domain, and class of the attribute is always relatively stable: considering the internal structure of the class, classes with the same attribute may be similar, and the same class may have similar attributes. Considering the internal structure of the attribute, it is considered that the definition domain and value domain of the same attribute may be similar, and the attributes with the same definition domain and value domain may be similar. Therefore, if the ontology contains rich internal structure information, the internal structure similarity between entities can be calculated. The key to judging the reliability of the internal structure similarity lies in the richness of the internal structure information in the ontology and the difference in the detailed description of the internal structure information of the two to-be-matched ontologies.

This section determines the reliability of the similarity method based on the internal structure by examining the richness of the internal structure, so as to lay the foundation for determining the weight of the similarity of the internal structure in the calculation of the comprehensive similarity of the structure.

The internal features of each pair of matched nodes obtained in the initial matching stage are analyzed. Different from calculating the external features of nodes, it is necessary to distinguish between classification and attribute nodes, because their internal structure information is different, so different methods are adopted when examining their information richness.

We use a vector to represent these internal features of the two classes and use the cosine similarity to calculate the internal feature similarity of the class nodes:

(7) $$\begin{array}{c} {\text{Sim}}_{I,C}\left(e_{1i},e_{2j}\right)=\text{Cos}\left(A_{1i,C}\right)•\text{Cos}\left(B_{2j,C}\right). \end{array}$$

For the internal features of the attribute node pair, the main test is whether the attribute has domain and range, which is also represented by a vector, and the cosine similarity is used to calculate the internal feature similarity of the attribute node:

(8) $$\begin{array}{c} {\text{Sim}}_{I,P}\left(e_{1i},e_{2j}\right)=\frac{A_{1i,P}•B_{2j,P}}{\left|A_{1i,P}-B_{2j,P}\right|}. \end{array}$$

### 2.5. Phoneme Segmentation

The construction of a neural network training model requires a large amount of labeled data, and it is usually difficult to obtain a large training set and test set. Usually, the available labels are text labels of isolated words or continuous sentences. The spectrogram corresponding to a specific word is sent to the neural network, and the trained model can output the posterior probability of each word during the test. However, due to the large number of English words, it is obviously unrealistic to obtain labeled data for all words and exhaustively list them all. However, all words are composed of phonemes after all, and phonemes can be exhausted. Different phonemes will have different performances on the spectrogram. Using phonemes as label units can train robustness in a limited training set. Therefore, this paper intends to use the phoneme as the label unit and use the edge detection method to segment the spectrogram of the isolated word to simulate the forced alignment processing of the speech spectrum signal by GMM-HMM.

Because the broadband spectrogram has better time resolution and can clearly distinguish the trend of the formants and the colors of different structures, the broadband spectrogram is used for phoneme segmentation processing. The process of spectrogram phoneme segmentation can be regarded as the process of finding the start and end edges of each phoneme from a segment of energy grayscale spectrogram. The introduced deformation function is as follows:

(9) $$\begin{array}{c} F\left(t\right)=\underset{f⟶F}{\prod }\left[E\left(F,t\right)-\left|E\left(F,t^{\prime }\right)\right|\right], \end{array}$$

(10) $$\begin{array}{c} E\left(F,t^{\prime }\right)=\underset{t^{\prime }⟶t+L}{\text{Max}}\left|\underset{f⟶F}{\prod }E\left(F,t^{\prime }\right)\right|. \end{array}$$

Among them, *F*(*t*) is the final deformation function, and *E*(*f*, *t*) represents the energy value (that is, the gray value) when the time is *t* and the frequency is *f*. When there is a large change in the energy distribution, *F*(*t*) will produce a peak. When the peak exceeds a threshold, the current position can be regarded as the end of the previous segment and the beginning of the next new segment.

After judging the peak value of the deformation function, each phoneme boundary can be basically divided, and the calculation speed is relatively fast. Then, the overall average energy distribution can be used to correct the situation of missing edges, and the context information of the phoneme features can be used to eliminate redundant edges. The alignment strategy adopted in this paper is as follows.

When the number of fragments segmented is the same as the number of phonemes in the corresponding word, they are aligned in chronological order.

When the number of fragments is different from the number of phonemes in the word, for example, the number of fragments is less than the number of phoneme labels by *n*, the first *n* fragments with the longest length are temporarily divided into half. This article categorizes the entire word into a separate file location for manual adjustment.

### 2.6. Pronunciation Evaluation Model Based on Convolutional Neural Network

A convolutional neural network is essentially a mathematical model based on supervised learning. It consists of multiple convolutional layers and pooling layers that alternately form the front end of the entire network for feature extraction and multiple fully connected layers at the back end for global integration and transformation of the extracted local features. The output is dynamically adjusted for different tasks. After the image preprocessing in the previous step, we obtained the spectrogram feature input with a large effective area ratio and the labeled data specific to the phoneme.

With the continuous alternation of convolutional layers and pooling layers, the expressive power of CNN is also significantly enhanced. In addition, through a certain number of convolution operations, the pooling layer can obtain information on different temporal dimensions of speech, which enhances the robustness of the model.

The front end of the entire network is composed of a convolution layer and a pooling layer. The convolution layer obtains the local information of the input features through the convolution kernel and then passes it to the pooling layer for generalization. The local information in the feature can be better obtained by alternately processing the feature twice, and then, the fully connected layer at the back end performs global information integration, and the entire network finally outputs the state category to which the current feature belongs.

Pooling reduces the input size while retaining the original important information, reduces the computational load of the model, and avoids the occurrence of overfitting by filtering the features of the information in the front layer.

By pooling the spectrogram, the influence of different speakers on the speech energy distribution is reduced, and the robustness of the model is enhanced, so that specific phonemes of nonspecific people can be more accurately identified.

#### 2.6.1. Model Structure

The implementation model trained in this paper uses an extended structure similar to Le Net-5. Among them, there are 2 convolutional layers, each convolutional layer is followed by a pooling layer, the convolutional layer and the pooling layer are combined, and the output after the convolution is directly used as the input of the pooling layer. The overall structure is shown in Figure 1.

Considering that the image input obtained after the aforementioned preprocessing is in the shape of long and narrow strips with the same height and uncertain width, but the input of the network model requires the same size of each input, and the current mature frameworks have a good initial value for square image input. Parameter support, that is, a relatively stable prediction result, can be achieved without a very large training set.

Therefore, we convert the feature input image to a square size of 256∗256 and keep the aspect ratio of the original image and fill it into the square and fill the unfilled places with 0 values.

Considering that the final output is the probability that the image belongs to each phoneme, the overall number of categories is large, and each phoneme is mutually exclusive, so softmax is finally used as the classifier.

The entire model is an ordered concatenated structure. After the model structure is confirmed, the optimization algorithm for parameter tuning needs to be determined. The stochastic gradient descent algorithm is used here, and the loss function and other elements need to be defined in advance. After the model structure is completed, the next step is the training of the model. After several iterations, the parameters are optimized until the model recognition accuracy tends to be stable. Before starting training, it is necessary to determine the number of training steps, batches, and the total number of iterations. Generally, an empirical value is used as the initial value.

#### 2.6.2. Dropout Method

Deep convolutional neural networks need to train many parameters, especially in the fully connected layer. If there is very little training data during training, it is easy to cause overfitting. To solve this problem, the model training process can usually be monitored with an additional validation set, and the iterations stopped early.

At each training time, each neuron has a certain probability to be temporarily removed, so part of the feature detectors will stop working, and their parameters will not participate in the update, and they will have a certain probability when waiting for the next iteration, which can weaken the joint adaptability between neuron nodes and improve the generalization ability of the network and the robustness of prediction.

Due to the computational characteristics of dropout, the model obtained after each dropout is a subset of the original model, and all iterations can be regarded as the average calculation of the results of different subnetworks. The formula of the normal neural network model can be expressed as follows:

(11) $$\begin{array}{c} z_{i,\left(l+1\right)}=w_{i,\left(l+1\right)}y_{l}+b_{l+1,i}, \end{array}$$

(12) $$\begin{array}{c} y_{i,\left(l+1\right)}=w_{i,\left(l+1\right)}•f\left[z_{i,\left(l+1\right)}\right]. \end{array}$$

After dropout, each unit of the network needs to go through a probabilistic process.

When adding dropout for prediction, each neuron needs to be premultiplied by a Bernoulli function, which represents a random 0-1 vector with probability. After the calculation, about *p*∗100 percent of the cell values will be set to 0. During the testing phase, the weight of the test value is also multiplied by the probability.

When the hidden layer nodes are multiplied by the function of probability value *p* = 0.5, dropout randomly generates the most network structures, and the final effect is also the best. When using dropout in this article, the probability value used is also 0.5.

## 3. Results

### 3.1. Validity Analysis Based on Discrimination

Based on the validity of the discriminativeness of the indicators, two factors are investigated. One is the “intraclass distance.” The index values of the same class are close to each other, indicating that the index is effective; the second is the “interclass distance”; the index values between different classes are different. In this section, the effectiveness of speech emotion indicators is reflected by observing the discriminativeness of speech emotion evaluation results under different manual evaluation results. “Intraclass distance” observes the variance of speech emotion evaluation results under the same manual rating, and “interclass distance” observes the mean of speech emotion evaluation results under different manual ratings, and one-way ANOVA is used to verify the statistical significance of the mean difference.

Figure 2 shows the variance of speech emotion evaluation results in different artificial ratings, corresponding to the four emotions of happiness, sadness, anger, and surprise, respectively. The variance of the speech emotion evaluation results of the same manual rating is small, and the variance of different ratings is stable, indicating that the speech emotion index is effective. By observing Figure 2, it can be seen that the variance fluctuates in a relatively small range, indicating that the data within the four levels is relatively stable.

There is a difference in the “interclass spacing,” and the clustering between classes is displayed, indicating that the indicator is effective. That is to say, the speech emotion evaluation results of different ratings are different, and the rules are consistent with the manual evaluation results, indicating that the speech emotion evaluation results are valid. The speech emotion evaluation results show the same trend as the manual evaluation; that is, the lower the manual evaluation, the lower the speech emotion evaluation result.  Table 1 lists the average number of speech emotion evaluation results under different manual ratings, and it can be seen that different ratings can be distinguished. However, whether this difference in the mean of different manual ratings is essential or random, this paper uses one-way analysis of variance to test. By observing the *p* values in the data result table, it can be seen that the *p* values under all 4 emotions are less than 0.05, indicating that the difference between the pronunciation quality levels of different speech emotions is statistically significant.

### 3.2. Validity Analysis Based on Comprehensive Evaluation Reliability

Another way to analyze the validity of the indicators is to compare the performance before and after the indicators are added to the model. In this paper, the performance is reflected by the human-machine evaluation reliability. Three test values of exact agreement rate, adjacent agreement rate, and Pearson correlation coefficient are used to analyze the reliability of human-machine evaluation.

In this paper, the ID3 algorithm is used to construct a decision tree that includes speech emotion indicators and those that do not include speech emotion indicators and conducts a comprehensive evaluation of computer automatic pronunciation quality. The results of the two evaluations are shown in Figure 3. It can be seen from Figure 3 that after the speech emotion index is added to the comprehensive evaluation model of pronunciation quality, the precise agreement rate, adjacent agreement rate, and correlation coefficient are all improved, but the improvement extent is different. Among them, the Pearson correlation coefficient is improved from positive correlation to strong positive correlation, and the improvement of the exact agreement rate is greater than that of the adjacent agreement rate.

Based on discrimination and the validity analysis results based on comprehensive evaluation reliability, the speech emotion pronunciation quality evaluation method designed in this paper is effective.

### 3.3. Reliability Analysis of Human-Machine Evaluation of Pronunciation Quality

It can be seen from Figure 4 that the deviation of the number of samples in each score segment between the manual rating and the machine rating of the test set is kept within a reasonable range. From the overall observation, the distribution of this rating sample conforms to the performance distribution characteristics of the general test. Observing the distribution and data volume, the machine rating meets the approximate requirements for the test rating. However, from a microscopic observation, human ratings and machine ratings still show differences. Human-rated scores are relatively high, and machine-rated ratings are “stricter.” The error between human rating and machine rating is shown in Figure 5.

From Table 2, we can see the specific data to observe the data of machine ratings corresponding to manual ratings under different ratings. In a separate analysis of surprise sentiment data, it was found that human evaluations were high, 1-level data sets were more, and machine ratings were more moderate, as shown in Table 3. The role of this part of the data also leads to a left-shifted distribution of the overall machine ratings. When analyzing the validity of speech emotion evaluation, the problem has been described in the previous article. The machine evaluation model is not effective in distinguishing data with similar characteristics, so the classification confidence output value is low, and the manual rating is used in the surprise emotion corpus. The rating adopts a subjective high-scoring strategy.

## 4. Discussion

### 4.1. Ontology Heterogeneity and Ontology Matching

With the explosive growth of Semantic Web information, more and more ontologies exist and are applied on the Internet [16, 17]. The creation and use of ontologies are subjective, autonomous, and distributed, which increases the number of ontologies that express similar meanings. Even in the same field, there are often a large number of ontologies, and the content they describe is often overlapping or related in semantics, but there are differences in the language and representation model of the ontology used [18]. This phenomenon is called ontology heterogeneity. There are various forms of ontology heterogeneity, which can be generally divided into two levels.

The first level is the heterogeneity at the language level, which means that the metalanguage used to describe the ontology is heterogeneous, which includes not only the mismatch between the grammar of the ontology language and the language primitives used but also the definition of classes. The heterogeneity of the semantic layer is divided into four categories: grammatical heterogeneity, logical representation heterogeneity, semantic heterogeneity of primitives, and language expression ability heterogeneity.

The second level of ontology heterogeneity is the heterogeneity on the model layer, which refers to the mismatch caused by different ontology modeling methods, including the conceptualization abstraction heterogeneity of different modelers and the same concept or relationship [19, 20]. The mismatch of the model layer is divided into two categories: conceptual heterogeneity and interpretation heterogeneity [21].

Conceptualized heterogeneity is divided into scope heterogeneity and model coverage heterogeneity. Concept scope means that concepts with the same name often have different meanings in different fields; different modelers often divide concepts differently in the modeling process due to different domain requirements or subjective understandings [22–24]. Model coverage refers to the difference in the knowledge scope and level of detail described by different ontologies. The differences in model coverage are further divided into the breadth of the model, the granularity of the model, and the viewpoint of ontology modeling [25].

Interpretation heterogeneity is divided into model style heterogeneity and modelling term heterogeneity. The heterogeneity of modeling style includes the heterogeneity of paradigm and the heterogeneity of concept description [26]. Paradigm heterogeneity means that different paradigms can be used to represent the same concept. Concept description heterogeneity means that in ontology modeling, there are several options for modeling the same concept [27–29]. For example, to distinguish two classes, either use an appropriate property or reference a separate class. Modeling term heterogeneity includes three types of heterogeneity: synonymous term, homomorphic term, and encoding format. The synonymous term heterogeneity refers to concepts that have the same meaning in different ontologies and are often represented by different names due to the habit of the modeler [30, 31].

### 4.2. The Theoretical Model of Language Testing

American applied linguists have proposed a new communicative language ability test model, which has had a wide-ranging impact in the British and American testing circles and is considered to be a “milestone in the history of language testing” [32]. He believes that there is an intrinsic link between the research and development of language learning and language teaching and language testing. The two influence each other and promote each other. He also believes that a learner's language ability should have a broader meaning. In addition to the mastery of the knowledge of language systems, it must also include the mastery of the context in which the language is used other than sentences [28, 33, 34]. Language communication is not just a simple information transfer, but a dynamic interaction between situations, language users, and discourse.

With the improvement of test theory, the development of computer technology, and the application of multimedia technology, more and more computers are used in language testing, and the methods and means of language testing begin to undergo fundamental changes [16]. Because computers have the characteristics of large storage capacity, fast processing speed, strong analysis ability and timely information feedback, computer-aided teaching, and computerized testing methods have gradually become popular, and network learning environments and testing methods have also begun to develop [35]. Many aspects of language learning and language testing have been developed through computer-assisted instruction and the use of computerized testing methods. There are also some problems that should be paid attention to in computer language testing.

First, the development and implementation of an effective computer-aided test system require a lot of time and effort, and its effective application also depends on the available computer hardware and software. Second, computer-assisted language testing is also limited by screen size. Although most computer systems today have overcome the 80-character limit of 25 lines a few years ago, the material that can be displayed on a single screen is still very limited [36]. Third, the use of computers to analyze students' answers to quizzes is still limited by two aspects. First, the ability to use computer hardware to recognize text is a new technology, which is expensive; second, the application of computers for natural language analysis is not enough. The analysis that can be carried out is mostly the results of artificial intelligence research and has not yet reached the practical stage. Fourth, a perfect computer adaptive test requires high research and development costs and a lot of time, and the development of testing technology is still in a bottleneck period.

As the computer-based personalized teaching method enters the field of English teaching, the English test method will gradually transition from the current manual test to the computer test. The development of computer network is also the development of network testing. Some exams are already administered through a computer network.

Its advantages mainly include flexibility in time and space and low cost. The main disadvantage is that the confidentiality of the test questions is not good. In addition, the recent emergence of electronic raters and “telephone tests” is also the application of computer technology in language testing. The development and utilization of E-rater reflect the development trend in the field of testing, that is, the combination of computer technology, cognitive science theory, and artificial intelligence technology to explore the process of people's problem solving, which has far-reaching significance for improving the reliability of test evaluation.

### 4.3. Validity and Reliability of the Oral English Test

The validity of a language test refers to whether the test achieves the intended test intent [37]. If a set of questions in the test involves something other than the purpose of the test, then the validity of the set is very low. The ultimate purpose of language learning is to communicate, so test scoring should focus on judging candidates' ability to communicate effectively, that is, the accuracy of language, the fluency of language used, and the appropriateness of the language used to the context. In the specific scoring process, the spoken language scoring system is roughly evaluated from three aspects: the accuracy of language and the breadth of language application (coverage), the length and coherence of discourse, and the flexibility of language and the adaptability of language to context [21, 38].

In order to ensure the scientificity and validity of the systematic test questions, a large number of test samples should be organized in advance, sampling tests should be conducted, and the validity of the test questions should be corrected. Some technical parameters of the subject can be realized. The use of computer technology must be able to conveniently complete the storage, expansion, and modification of the test questions, and the test papers can be automatically generated according to a certain mode.

Test reliability is essential for any valid test, and test reliability is the consistency, reliability, and stability of test scores. If a test has high reliability, no matter how many times the test is administered to the same group of students under any circumstances, the students' scores on each test should be consistent and represent the true ability of the test taker [39].

Oral exams deal with language in a variety of ways, and there are many aspects to be examined in scoring, so a standard should be set first. The subject uses the analytical method to compare and score each word and even phoneme, including intonation, rhythm, speed, volume and pitch, and score subitems [40]. After applying the scoring template, the final similarity score is obtained.

Some scholars have tried to verify the validity and reliability [41]. After reviewing the factors that affect the scoring and the current methods that mainly focus on the spoken language scoring, a method for objective scoring of the spoken language was proposed [42]. After defining it in a theoretical and operational sense, an experiment was carried out. This is an empirical study based on a speech corpus. A total of 25 quantitative indicators were extracted from the PETS Level 3 Oral Test Analytical Score [43]. The data extracted from the speech and written text of 30 test takers were then input into SPSS for stepwise linear regression analysis, resulting in a corresponding model. These models were able to identify most of the variance variation in speaking scores.

## 5. Conclusion

In this paper, when the model is trained, it is forced to have a small sample of data, and the mean of the results of each model is calculated in the way of bagging. The experimental data results show that the variance of speech emotion evaluation results within the same rating is low and stable; the mean value of speech emotion evaluation results under different manual ratings, and the manual rating results show the same trend, and the data differences between different ratings are essential. The computer automatic evaluation performance of the comprehensive evaluation results of pronunciation quality has been improved. Intonation, speech rate, rhythm, intonation, and emotion are used together as indicators for comprehensive evaluation of pronunciation quality in this paper. The traditional linear mapping method is not suitable for the comprehensive evaluation of pronunciation quality of multi-index fusion, because the corpus data used in this paper adopts the overall scoring mode. After simulating and abstracting the overall scoring process, this paper believes that the scoring process is similar to the binary tree structure, so this paper uses a decision tree to build an evaluation method. Using the ID3 algorithm, considering the information gain of each index, a multi-index comprehensive evaluation decision tree is constructed. The machine evaluation shows that the accurate consistency rate of human-machine evaluation reaches 93%, the adjacent consistency rate is 94.7%, and the correlation coefficient is 0.89, which shows that the evaluation method in this paper is credible.

## Figures and Tables

**Figure 1:** Structure diagram of the CNN model used in this paper.

**Figure 2:** Emotional machine evaluation variance of different human evaluation levels.

**Figure 3:** Comparison of the reliability of human-machine evaluation between the two groups.

**Figure 4:** Distribution of human-machine ratings.

**Figure 5:** Error between human rating and machine rating.

**Table 1:** Mean value of speech emotion evaluation results.

Human rating	A	B	C	D	*F* value	*p* value
Happy	0.378	0.331	0.302	0.271	6	0
Sad	0.360	0.331	0.310	0.264	6.9	0
Angry	0.371	0.334	0.303	0.275	7.2	0
Surprise	0.321	0.311	0.301	0.296	6.1	0

**Table 2:** Number of paired samples for human-machine rating.

Human review/machine review	Level 1	Level 2	Level 3	Level 4
Level 1	157	62	47	2
Level 2	27	214	48	25
Level 3	1	34	216	58
Level 4	2	4	28	123

**Table 3:** The number of comparative samples of human-machine rating of surprise corpus.

Human review/machine review	Level 1	Level 2	Level 3	Level 4
Level 1	72	43	42	2
Level 2	1	53	37	1
Level 3	2	15	27	12
Level 4	1	7	17	26

## Data Availability

The data used to support the findings of this study are available from the corresponding author upon request.

## References

[1] Shaqra F. A., Duwairi R., Al-Ayyoub M. (2019). Recognizing emotion from speech based on age and gender using hierarchical models. *Procedia Comput. Sci.*.

[2] Thongsuwan S., Jaiyen S., Padcharoen A., Agarwal P. (2021). ConvXGB: a new deep learning model for classification problems based on CNN and XGBoost. *Nuclear Engineering and Technology*.

[3] Arora V., Lahiri A., Reetz H. (2018). Phonological feature-based speech recognition system for pronunciation training in non-native language learning. *The Journal of the Acoustical Society of America*.

[4] Weldegebriel H. T., Liu H., Haq A. U., Bugingo E., Zhang D. (2020). A new hybrid convolutional neural network and eXtreme gradient boosting classifier for recognizing handwritten Ethiopian characters. *IEEE Access*.

[5] Klaylat S., Osman Z., Hamandi L., Zantout R. (2018). Emotion recognition in Arabic speech. *Analog Integrated Circuits and Signal Processing*.

[6] Wang F., Li Z., He F., Wang R., Yu W., Nie F. (2019). Feature learning viewpoint of AdaBoost and a new algorithm. *IEEE Access*.

[7] Cámara-Arenas E. (2014). The NCM and the reprogramming of latent phonological systems: a bilingual approach to the teaching of English sounds to Spanish students. *Procedia - Social and Behavioral Sciences*.

[8] Tejedor-Garcia C., Escudero-Mancebo D., Cardenoso-Payo V., Gonzalez-Ferreras C. (2020). Using challenges to enhance a learning game for pronunciation training of English as a second language. *IEEE Access*.

[9] Swain M., Routray A., Kabisatpathy P. (2018). Databases features and classifiers for speech emotion recognition: a review. *International Journal of Speech Technology*.

[10] Altwaijry N., Al-Turaiki I. (2020). Arabic handwriting recognition system using convolutional neural network. *Neural Computing and Applications*.

[11] Pyshkin E., Blake J., Lamtev A., Lezhenin I., Zhuikov A., Bogach N. (2019). Prosody training mobile application: early design assessment and lessons learned. *Proc. 10th IEEE Int. Conf. Intell. Data Acquisition Adv. Comput. Systems: Technol. Appl. (IDAACS)*.

[12] O’Brien M. G., Derwing T. M., Cucchiarini C. (2022). Directions for the future of technology in pronunciation research and teaching. *J. Second Lang. Pronunciation*.

[13] Badshah A. M., Rahim B. N., Ullah N. (2019). Deep features-based speech emotion recognition for smart affective services. *Multimedia Tools and Applications*.

[14] Chen C.-H., Liu J.-H., Shou W.-C. (2018). How competition in a game-based science learning environment influences students’ learning achievement flow experience and learning behavioral patterns. *Journal of Educational Technology & Society*.

[15] Munteanu C., Molyneaux H., Maitland J. (2014). Hidden in plain sight: low-literacy adults in a developed country overcoming social and educational challenges through mobile learning support tools. *Personal and Ubiquitous Computing*.

[16] Liakin D., Cardoso W., Liakina N. (2017). The pedagogical use of mobile speech synthesis (TTS): focus on French liaison. *Computer Assisted Language Learning*.

[17] Meftah A. H., Alotaibi Y. A., Selouani S.-A. (2018). Evaluation of an Arabic speech corpus of emotions: a perceptual and statistical analysis. *IEEE Access*.

[18] Kibishi H., Hirabayashi K., Nakagawa S. (2015). A statistical method of evaluating the pronunciation proficiency/intelligibility of English presentations by Japanese speakers. *ReCALL*.

[19] Boufenar C., Kerboua A., Batouche M. (2018). Investigation on deep learning for off-line handwritten Arabic character recognition. *Cognitive Systems Research*.

[20] Mustafa M. B., Yusoof M. A. M., Don Z. M., Malekzadeh M. (2018). Speech emotion recognition research: an analysis of research focus. *International Journal of Speech Technology*.

[21] Eksi G. Y., Yesilcinar S. (2016). An investigation of the effectiveness of online text-to-speech tools in improving EFL teacher trainees’ pronunciation. *English Language Teaching*.

[22] Alyahya H., Ben Ismail M. M., Al-Salman A. (2020). Deep ensemble neural networks for recognizing isolated Arabic handwritten characters. *Accent. Trans. Image Process. Comput. Vis.*.

[23] Abraham B., Umesh S. (2017). An automated technique to generate phone-to-articulatory label mapping. *Speech Communication*.

[24] Palo H. K., Mohanty M. N. (2018). Wavelet based feature combination for recognition of emotions. *Ain Shams Engineering Journal*.

[25] Lee J., Jang J., Plonsky L. (2015). The effectiveness of second language pronunciation instruction: a meta-analysis. *Applied Linguistics*.

[26] Sepehr S., Head M. (2018). Understanding the role of competition in video gameplay satisfaction. *Information Management*.

[27] de Vries B. W. F. P., Cucchiarini C., Strik H., van Hout R. (2019). Spoken grammar practice in CALL: the effect of corrective feedback and education level in adult L2 learning. *Language Teaching Research*.

[28] Thomson R. I., Derwing T. M. (2015). The effectiveness of L2 pronunciation instruction: a narrative review. *Applied Linguistics*.

[29] Li K., Qian X., Meng H. (2017). Mispronunciation detection and diagnosis in l2 English speech using multidistribution deep neural networks. *IEEE/ACM Trans. Audio Speech Lang. Process.*.

[30] Balaha H. M., Ali H. A., Saraya M., Badawy M. (2020). A new Arabic handwritten character recognition deep learning system (AHCR-DLS). *Neural Computing and Applications*.

[31] Sailer M., Hense J. U., Mayr S. K., Mandl H. (2017). How gamification motivates: an experimental study of the effects of specific game design elements on psychological need satisfaction. *Computers in Human Behavior*.

[32] Vathsala M., Holi G. (2020). RNN based machine translation and transliteration for Twitter data. *International Journal of Speech Technology*.

[33] Jiang P., Fu H., Tao H. (2019). Speech emotion recognition using deep convolutional neural network and simple recurrent unit. *Engineering Letters*.

[34] Jalalvand S., Negri M., Falavigna D., Matassoni M., Turchi M. (2018). Automatic quality estimation for ASR system combination. *Computer Speech & Language*.

[35] Nagle C. (2018). Motivation, comprehensibility, and accentedness in L2 Spanish: investigating motivation as a time-varying predictor of pronunciation development. *The Modern Language Journal*.

[36] Cagiltay N. E., Ozcelik E., Ozcelik N. S. (2015). The effect of competition on learning in games. *Computers in Education*.

[37] Akhter M. P., Jiangbin Z., Naqvi I. R., Abdelmajeed M., Sadiq M. T. (2020). Automatic detection of offensive language for Urdu and roman Urdu. *IEEE Access*.

[38] Khan W., Daud A., Khan K. (2019). Part of speech tagging in Urdu: comparison of machine and deep learning approaches. *IEEE Access*.

[39] Huynh D., Iida H. (2017). An analysis of winning streak’s effects in language course of ‘Duolingo. *Asia–Pacific J. Inf. Technol. Multimedia*.

[40] Yüksel M., Gündüz B. (2018). Long term average speech spectra of Turkish. *Logopedics, Phoniatrics, Vocology*.

[41] Gaffary Y., Argelaguet F., Marchal M. (2018). Toward haptic communication: tactile alphabets based on fingertip skin stretch. *IEEE Transactions on Haptics*.

[42] Shams M., Elsonbaty A., ElSawy W. (2020). Arabic handwritten character recognition based on convolution neural networks and support vector machine. *International Journal of Advanced Computer Science and Applications*.

[43] Ehsan T., Hussain S. (2019). Analysis of experiments on statistical and neural parsing for a morphologically rich and free word order language Urdu. *IEEE Access*.

